The article "Identifying miRNAs Associated with the Progression of Keloid through mRNA-miRNA Network Analysis and Validating the Targets of miR-29a-3p in Keloid Fibroblasts" was published in 2022. Journal: Biomed Res Int.

# Identifying miRNAs Associated with the Progression of Keloid through mRNA-miRNA Network Analysis and Validating the Targets of miR-29a-3p in Keloid Fibroblasts

**DOI:** 10.1155/2022/6487989

**Published:** 2022-07-13

**Authors:** Yan He, Zexin Zhang, Bin Yin, Shu Li, Peng Wang, Junhong Lan, Wenqin Lian, Chiyu Jia

**Affiliations:** ^1^School of Medicine, Xiamen University, Xiamen, China; ^2^Department of Burns and Plastic and Wound Repair Surgery, Xiang'an Hospital of Xiamen University, School of Medicine, Xiamen University, Xiamen, Fujian, China

## Abstract

**Background:**

Keloid has brought great trouble to people and currently has no uniformly successful treatment. It is urgent to find new targets to effectively prevent the progress of keloid. The current research mainly identifies the differentially expressed genes (DEGs) in keloid through high-throughput sequencing technology and bioinformatics analysis technology, to screen new therapeutic targets and potential biomarkers. However, due to the different samples, different control groups, and small sample sizes, the sequencing results obtained from different studies are quite different and lack reliability. It is necessary to analyze the existing datasets in a reasonable way.

**Methods:**

Datasets about keloid were filtered in Gene Expression Omnibus (GEO) and ArrayExpress databases according to the inclusion and exclusion criteria. The discovery datasets were used for summarizing significant DEGs, and the validation datasets were to validate the mRNA and miRNA expression levels. The Encyclopedia of RNA Interactomes (ENCORI) online platform was used to predict the interactions between miRNAs and their target mRNAs. Protein-protein interaction network (PPI network) analysis and functional enrichment analysis were conducted. miRNA-mRNA network was established by Cytoscape software and verified in keloid tissue (*n* = 8) by RT-qPCR. miR-29a-3p mimic and inhibitor were transfected into keloid fibroblasts (KFs) to preliminary verify its targets, the prognostic value of which was estimated by the receiver operating characteristic (ROC) curve.

**Results:**

A total of 6 datasets involving 20 patients were included. 15 miRNAs and 12 target mRNAs were identified as potential biomarkers for keloid patients. The RT-qPCR results showed that miR-29a-3p, miR-92a-3p, and miR-143-3p were downregulated, and all their target mRNAs were upregulated in keloid tissue (*P* < 0.05). The expression of COL1A1, COL1A2, COL3A1, COL5A1, and COL5A2 decreased when miR-29a-3p was overexpressed but increased when miR-29a-3p was knocked down (*P* < 0.05). And these genes had a good performance in the diagnosis of keloid, especially when using keloid nonlesional skin or normal scar tissues as controls.

The article "Identifying miRNAs Associated with the Progression of Keloid through mRNA-miRNA Network Analysis and Validating the Targets of miR-29a-3p in Keloid Fibroblasts" was published in 2022. Journal: Biomed Res Int.

**Conclusion:**

The miRNA-mRNA network, especially miR-29a-3p and its targets, may provide insights into the underlying pathogenesis of keloid and serve as potential biomarkers for keloid treatment.

## 1. Introduction

Keloid is a complex fibroproliferative disease similar to the benign tumor growing outside the edge of the original wound, which can cause skin dysfunction and aesthetic deformity by invading adjacent normal tissues [1]. In addition, a cross-sectional survey on the burden of keloid shows that keloid has caused serious damage to the emotional health of patients [2]. In a word, keloids pose a great threat to people's physical and mental health, but the underlying pathogenesis of keloid formation remains to be elucidated, and the treatments for keloid are not satisfactory (including triamcinolone acetonide injection, surgical resection, and radiotherapy) [3, 4]. Therefore, it is urgent to seek effective biomarkers of keloid, which can further reveal the molecular mechanism of keloid formation and provide new insights for the development of treatment methods.

miRNA is a kind of noncoding single-stranded RNA with a length of about 22 nucleotides. It can bind hundreds of target genes and regulate their expression. A large number of studies have confirmed that the miRNA-mRNA axis affects the development of keloid by regulating cell proliferation, apoptosis, migration, invasion, and collagen synthesis [5]. Therefore, miRNAs that play an important role in the development of keloid may become new targets for the treatment of keloid [6].

The current research identifies abnormally expressed genes to screen new therapeutic targets and potential biomarkers mainly through high-throughput sequencing technology and bioinformatics analysis technology [7–9]. However, the sequencing results obtained from different studies are quite different. There are three main reasons: (1) the high cost of high-throughput sequencing technology makes it difficult to sequence large-scale samples. (2) The samples used for detecting are different (including keloid tissue, keloid fibroblast, and keloid keratinocyte). (3) The source of normal skin used as control is different (including normal skin of keloid patients, normal skin of healthy people, and foreskin). Therefore, to obtain reliable results, it is necessary to analyze the existing datasets in a reasonable way.

In our study, datasets about keloid were filtered in Gene Expression Omnibus (GEO) and ArrayExpress databases according to the inclusion and exclusion criteria. Four datasets (GSE92566, GSE83286, GSE158395, and GSE190626) were screened and treated as discovery datasets for summarizing significantly differentially expressed genes (DEGs), and the other two datasets (GSE113619 and GSE113620) were served as validation datasets to validate the mRNA and miRNA expression levels. In addition, the functions of these DEGs were annotated by Gene Ontology (GO) enrichment analysis and Kyoto Encyclopedia of Genes and Genomes (KEGG) pathway enrichment analysis. Finally, a miRNA-mRNA network was established and verified in keloid tissue, and the targets of miR-29a-3p were preliminary verified in keloid fibroblasts (KFs). Our research was aimed at finding novel therapeutic targets for keloid.

The article "Identifying miRNAs Associated with the Progression of Keloid through mRNA-miRNA Network Analysis and Validating the Targets of miR-29a-3p in Keloid Fibroblasts" was published in 2022. Journal: Biomed Res Int.

## 2. Materials and Methods

### 2.1. Clinical Specimen Information and Fibroblast Culture

Lesional and nonlesional keloid skin samples were collected from patients undergoing keloid surgery in the Xiang'an Hospital affiliated with Xiamen University. The clinical specimen information is presented in Table 1. This experiment was conducted in accordance with the Declaration of Helsinki and with the approval of the Medical Ethics Committee of Xiang'an Hospital Affiliated with Xiamen University and informed patient consent in writing.

The primary fibroblasts were successfully isolated based on the previously reported procedures. Briefly, we removed the epidermis and fat of the skin specimen. The dermal tissue was cut into 5 mm^2^ explants and was evenly distributed in the sterile Petri dish. The explants were incubated in Dulbecco's Modified Eagle Medium supplemented with 10% fetal bovine serum and 2% penicillin-streptomycin in an atmosphere of 5% carbon dioxide for the primary and subsequent cultures. The KFs at passages 3-5 were carried out to subsequent experiments.

### 2.2. Datasets

The Gene Expression Omnibus (GEO) (https://www.ncbi.nlm.nih.gov/geo/) and ArrayExpress (https://www.ebi.ac.uk/arrayexpress/) databases were searched to identify relevant transcriptomic profiling datasets. Datasets containing keloid transcriptomic profiling in Homo sapiens were potentially eligible. Datasets were excluded if they were not assaying keloid tissue samples, not measuring mRNA or miRNA, and not taking the nonlesional skin of keloid patients themselves as the control group. Furthermore, datasets that did not contain complete expression data were also excluded. Additional datasets could be added by manual search of the reference of included studies. The data of this part is obtained from the public database, so it is not necessary to obtain the patient's informed consent and ethical review.

### 2.3. Data Processing

R software (version 4.0.3) was used to convert the ID of datasets, and probes with missing gene symbols were excluded. The “LIMMA” software package was used to analyze the DEGs in the datasets (adj.*P*.value < 0.05, |logFC| > 1). These DEGs were visualized by volcano plots. We screened common differentially expressed genes (co-DEGs) existing in at least 3 discovery datasets and divided co-DEGs into two groups, namely, co-up DEGs and co-down DEGs.

The article "Identifying miRNAs Associated with the Progression of Keloid through mRNA-miRNA Network Analysis and Validating the Targets of miR-29a-3p in Keloid Fibroblasts" was published in 2022. Journal: Biomed Res Int.

### 2.4. Functional Enrichment Analysis

Gene ontology (GO) enrichment analysis and Kyoto Encyclopedia of Genes and Genomes (KEGG) pathway enrichment analysis of co-up DEGs and co-down DEGs are carried out by using Bioinformatics online platform (http://www.bioinformatics.com.cn). GO enrichment analysis includes biological processes (BP), molecular functions (MF), and cellular components (CC).

### 2.5. Protein-Protein Interaction (PPI) Network Analysis and Identification of Hub Genes

STRING online platform (https://cn.string-db.org/) was used to construct the PPI network which was analyzed by Cytohubba (a plug-in of Cytoscape). The top 20 genes ranked by different methods were recorded, and genes recommended by at least 5 methods were selected. The expression level of these genes was further validated by the validation dataset. The validated co-DEGs were considered as Hub genes.

### 2.6. Establishment of miRNA-mRNA Network and Identification of Hub miRNA

Encyclopedia of RNA Interactomes (ENCORI) online platform [10] (https://starbase.sysu.edu.cn/index.php) was used to predict the miRNAs that regulated the Hub genes, and the list of miRNAs certified by at least three programs was downloaded. Select the miRNAs that can regulate at least 3 Hub genes, and these miRNAs were verified by validation dataset. The differentially expressed miRNAs were labeled Hub miRNA, and the miRNA-mRNA network was visualized by Cytoscape.

### 2.7. Quantitative Reverse Transcription PCR (RT-qPCR)

Total RNA was isolated using the Cell/Tissue Total RNA Kit (Yeasen, Shanghai, China) and reverse-transcribed using the RT reagent Kit (Takara, Dalian, China). RT-qPCR was performed using qPCR SYBR Green Master Mix (Yeasen, Shanghai, China) via a real-time PCR system (CFX96 Touch, Bio-Rad, USA). Primers for U6, miR-29a-3p, miR-92a-3p, and miR-143-3p were designed by Ruibo (Wuhan, China). The primer sequences were shown in Table 2. U6 and GAPDH were used as internal controls. The fold change in the relative gene expression to the control levels was determined using the standard 2−*ΔΔ*Ct method.

### 2.8. Cell Transfection

Mimics or inhibitors targeting miR-29a-3p and their respective blank controls were designed by Ruibo (Wuhan, China). To achieve better transfection efficiency, primary fibroblasts were seeded on 6-well plates in a conditioned medium without antibiotics and serum at a density of 5 × 10^4^ cells/mL. INTERFERin® (Polyplus, France) was applied to transfect these miRNAs into KFs according to the manufacturer's protocol. After transfection for 48 h, the expression of miR-29a-3p and the target genes were detected through qPCR.

The article "Identifying miRNAs Associated with the Progression of Keloid through mRNA-miRNA Network Analysis and Validating the Targets of miR-29a-3p in Keloid Fibroblasts" was published in 2022. Journal: Biomed Res Int.

### 2.9. Evaluation of Diagnostic Value

Different datasets were used to evaluate the diagnostic value of key genes. GSE92566, GSE83286, GSE158395, and GSE190626 were used to evaluate the diagnostic value of key genes between keloid lesional skin and nonlesional skin; GSE113619 was used to evaluate the diagnostic value of key genes between the normal skin from keloid-prone or normal individuals; GSE188952 was used to evaluate the diagnostic value of key genes between keloid tissue and hypertrophic scar or normal scar.

### 2.10. Statistical Analysis

All experiments were performed at least three times. The data are presented as the mean ± standard deviation (S.D.). Nominal variables were expressed as a count or as a percentage. The statistical comparisons between the groups were performed by paired Student's *t*-test or unpaired Student's *t*-test or one-way analysis of variance (ANOVA) using GraphPad Prism V. 9 (GraphPad Software, San Diego, CA, USA). *P* < 0.05 indicated a significant difference.

## 3. Results

### 3.1. Datasets Search and Characteristics of Included Datasets

A detailed overview of the selection process is shown in Figure 1. According to the inclusive and exclusive criteria, a total of 6 studies, including 20 patients, were enrolled in the analysis. In addition, a dataset (GSE188952) using hypertrophic scars and normal scars tissue as control was also included in the study to further evaluate the diagnostic value of key genes in keloid. The characteristics of the datasets included in the analysis are described in Table 3.

### 3.2. Identification of DEGs in Lesional and Nonlesional Skin of Keloid Patients

The “LIMMA” software package was used to analyze the DEGs in the discovery datasets. When adj.*P*.value < 0.05 and |logFC| > 1, 950 DEGs (462 upregulated and 488 downregulated), 524 DEGs (409 and 115), 1672 DEGs (696 and 976), and 1573 DEGs (856 and 717) between lesional and nonlesional skin were detected in GSE92566, GSE83286, GSE158395, and GSE190626 datasets, respectively (Figure 2). 493 co-DEGs (318 co-up DEGs and 175 co-down DEGs) exist simultaneously in at least 3 discovery datasets (Figures 3(a) and 3(b)). They are presented in Table 4.

### 3.3. Functional Enrichment Analysis

318 co-up DEGs and 175 co-down DEGs were analyzed by GO and KEGG analysis to explore their biological functions. It is worth noting that the 318 co-up DEGs in keloid are mainly related to the organization of extracellular matrix, extracellular structure, and collagen fibril, also involved in the development of bone, cartilage, and connective tissue (Figure 4(a)). The 175 co-down DEGs are mostly involved in sodium and potassium ion homeostasis and skin development (Figure 4(b)). In addition, the co-up DEGs and co-down DEGs are closely related to the focal adhesion (Figure 5(a)) and peroxisome proliferator-activated receptor (PPAR) signal pathways (Figure 5(b)) respectfully. A previous study had proved that increased transcriptional response to mechanical strain in keloid fibroblasts due to increased focal adhesion complex formation [11]. And Zhang et al. reported that troglitazone (PPAR-*γ* agonist) depressed transforming growth factor-*β*1-(TGF-*β*1-) stimulated collagen type I expression and collagen synthesis in keloid fibroblasts in a concentration-dependent manner [12]. These studies further confirmed the association between the focal adhesion and PPAR signal pathway and keloid.

The article "Identifying miRNAs Associated with the Progression of Keloid through mRNA-miRNA Network Analysis and Validating the Targets of miR-29a-3p in Keloid Fibroblasts" was published in 2022. Journal: Biomed Res Int.

### 3.4. Protein-Protein Interaction (PPI) Network Analysis and Identification of Hub Genes

The PPI network of 493 co-DEGs was constructed by STRING (Figure 6). The top 20 genes ranked by different methods of Cytohubba were presented in Table 5. 16 genes including COL1A1, COL1A2, COL3A1, COL5A1, COL5A2, COL6A1, COL6A2, COL6A3, COL11A1, FN1, POSTN, FBN1, TGFB3, LUM, SOX9, and BGN were recommended by at least 5 methods.

The expression level of the 16 genes was verified by the GSE113619 dataset. The results showed that the expression of 12 genes (Hub genes) significantly increased in the development of keloid (*P* < 0.05) while that of TGFB3, SOX9, and BGN did not change significantly (*P* > 0.05) (Figure 7). Unexpectedly, in the discovery datasets, the expression of FN1 was significantly upregulated in keloid but significantly downregulated in the GSE113619 dataset (Figure 7). Considering that the samples of GSE113619 were collected from the early stage of keloid formation and the samples of discovery datasets were mature keloid, this difference may be caused by different stages of keloid development, which needs more in-depth study to explore the characteristics at different stages of keloid.

### 3.5. Establishment of miRNA-mRNA Network and Identification of Hub miRNA

ENCORI was used to predict the miRNAs regulating the 12 Hub genes. Select the miRNAs that regulated at least 3 Hub genes, and the expression level of these miRNAs was verified by the GSE113620 dataset. The result showed that 15 miRNAs (Hub miRNA) were differentially expressed. Among them, miR-29a-3p, miR-92a-3p, and miR-143-3p were downregulated in the development of keloid, while the other 12 miRNAs were upregulated (*P* < 0.05) (Figure 8). We finally formed a miRNA-mRNA network composed of 12 mRNAs and 15 miRNAs by Cytoscape (Figure 9).

The article "Identifying miRNAs Associated with the Progression of Keloid through mRNA-miRNA Network Analysis and Validating the Targets of miR-29a-3p in Keloid Fibroblasts" was published in 2022. Journal: Biomed Res Int.

### 3.6. Identification of Quantitative Reverse Transcription PCR (RT-qPCR)

To further verify the miRNA-mRNA network, we detected the lesional and nonlesional keloid skin samples of 8 keloid patients by RT-qPCR. Considering that all Hub genes were upregulated and miRNA usually inhibits the expression of target genes, we mainly verified the 3 downregulated miRNAs and their upregulated targets. The results of RT-qPCR showed that miR-29a-3p, miR-92a-3p, and miR-143-3p showed a significant downregulation trend in keloid tissue, and the increase of their targets was also significant (Figure 10).

### 3.7. miR-29a-3p Regulated the Expression of COL1A1, COL1A2, COL3A1, COL5A1, and COL5A2 in KFs

The above results showed that miR-29a-3p was significantly downregulated in the development of keloid. More importantly, the miRNA-mRNA network showed that it can regulate the expression of 9 Hub genes (upregulated). Therefore, we speculated that miR-29a-3p plays a central role in Hub miRNA. Previous studies have confirmed that miR-29a-3p was significantly downregulated in keloid tissues and fibroblasts and can regulate the proliferation, apoptosis, migration, and invasion of KFs by targeting COL1A1 and COL3A1 [13, 14]. However, more potential targets for the role of miR-29a-3p remain to be clarified. To further verify the regulation of miR-29a-3p on the expression of these 9 Hub genes, we transfected miR-29a-3p mimic and inhibitor into KFs to detect the expression level of these Hub genes. RT-qPCR results showed that the expression of COL1A1, COL1A2, COL3A1, COL5A1, and COL5A2 decreased when miR-29a-3p was overexpressed but increased when miR-29a-3p was knocked down, indicating that these Hub genes may be potential targets for miR-29a-3p to regulate the biological behavior of KFs (Figure 11).

### 3.8. Diagnostic Value of COL1A1, COL1A2, COL3A1, COL5A1, and COL5A2 in Keloid

The diagnostic value of COL1A1, COL1A2, COL3A1, COL5A1, and COL5A2 between keloid and different control tissue was evaluated by different datasets. The results of the receiver operating characteristic (ROC) curve showed that when keloid nonlesional skin tissues were used as controls (GSE92566, GSE83286, GSE158395, and GSE190626), the AUC values of the 5 key genes in keloid were 1.000 (Figures 12(a)–12(d)). When the diagnostic value of these key genes were evaluated between the normal skin from keloid-prone or normal individuals (GSE113619), the AUC values of COL1A1, COL1A2, COL3A1, COL5A1, and COL5A2 in keloid were 0.650, 0.625, 0.575, 0.525, and 0.450, respectively (Figure 12(e)). When normal scar tissues were used as controls, the AUC values of the key genes in keloid were 1.000, 1.000, 1.000, 0.833, and 1.000, respectively (Figure 12(f)). When hypertrophic scar tissues were used as controls, the AUC values of the above genes were 1.000, 1.000, 0.900, 0.500, and 0.550, respectively (Figure 12(g)), indicating that these key genes had a good performance in the diagnosis of keloid, especially when using keloid nonlesional skin or normal scar tissues as controls. However, these genes cannot well distinguish the normal skin from keloid-prone or normal individuals.

The article "Identifying miRNAs Associated with the Progression of Keloid through mRNA-miRNA Network Analysis and Validating the Targets of miR-29a-3p in Keloid Fibroblasts" was published in 2022. Journal: Biomed Res Int.

## 4. Discussion

Keloid has brought great trouble to people and currently has no uniformly successful treatment [3]. Therefore, it is urgent to find new targets to effectively prevent the progress of keloid. In this study, a miRNA-mRNA network closely related to keloid was constructed through a comprehensive analysis of multiple datasets. miR-29a-3p was considered to be the real central miRNA through bioinformatics and molecular biology experiments. It was downregulated in keloid and can negatively regulate the expression of COL1A1, COL1A2, COL3A1, COL5A1, and COL5A2. It is suggested that miR-29a-3p plays an important role in the development of keloid and may become an effective target for the treatment of keloid.

The dysregulated expression of miR-29a-3p plays a role in a variety of fibrotic diseases including keloid. Zhang et al. found that the expression of miR-29a was significantly decreased in keloid tissues and fibroblasts (*n* = 9) compared with healthy controls (*n* = 6). They also found that the mRNA and protein levels of type I and type III collagen decreased in KFs with miR-29a overexpression and confirmed that it can directly regulate the expression of COL3A1 by luciferase gene reporting experiment [13]. Wang et al. confirmed that the expression of miR-29a in keloid tissue and fibroblasts (*n* = 80) was significantly lower than that in normal skin (*n* = 91) and could inhibit the viability, migration, invasion, and EMT of KFs while promoting its apoptosis. In addition, they proposed that miR-29a plays the above functions mainly by directly inhibiting the expression of COL1A1 [14]. Wu et al. found that miR-29a-3p was upregulated in hypertrophic scar (HS) tissue and fibroblasts compared with normal skin tissue and confirmed that miR-29a-3p inhibited the proliferation of hypertrophic scar fibroblasts (HSF) and the production of extracellular matrix (ECM) by directly targeting FRS2 [15]. Yuan et al. found that the expression level of miR-29a in mouse scar tissue was significantly downregulated compared with normal skin tissue and proposed that exosomes from miR-29a modified adipose mesenchymal stem cells could reduce excessive scar formation by inhibiting TGF- *β*2/Smad3 signal [16]. Nevertheless, more potential targets of miR-29a-3p have yet to be clarified.

The article "Identifying miRNAs Associated with the Progression of Keloid through mRNA-miRNA Network Analysis and Validating the Targets of miR-29a-3p in Keloid Fibroblasts" was published in 2022. Journal: Biomed Res Int.

In our study, the results of ENCORI prediction and RT-qPCR showed that miR-29a-3p can regulate the expression of COL1A1, COL1A2, COL3A1, COL5A1, and COL5A2, and these target genes were closely related to the development of keloid. Among them, COL1A1 and COL1A2 encode type I collagen and COL3A1 encodes type III collagen, the major components of the extracellular matrix in keloid tissue. Compared with normal skin, type I and III collagen deposition in keloid tissue increased significantly, and previous studies have confirmed that miR-29a-3p can regulate the biological behavior of KFs by directly targeting COL1A1 [14] and COL3A1 [13]. COL5A1 and COL5A2 are involved in encoding type V collagen, and its mutation is related to Ehlers-Danlos syndrome. Yokota et al. found that the expression of COL5A1 and COL5A2 was significantly increased in the early stage after acute ischemic heart injury, while the decrease of type V collagen leads to the contradictory increase of scar size after infarction [17]. However, there is no research report on the correlation between COL5A1 and COL5A2 expression and keloid so far.

In addition, Corrie et al. conducted a double-blinded, placebo-randomized, within-subject controlled clinical trial and found that remlarsen (a miR-29 mimic) repressed collagen expression and the development of fibroplasia in incisional skin wounds. They suggested that remlarsen may be an effective therapeutic to prevent the formation of a fibrotic scar (hypertrophic scar or keloid) or to prevent cutaneous fibrosis (such as scleroderma), which also provides strong human experimental evidence for the clinical application of miR-29a-3p in the treatment of keloid [18].

Except for miR-29a-3p, we also verified the expression level of 2 downregulated miRNA (miR-92a-3p and miR-143-3p). Mu et al. found that miR-143-3p was significantly downregulated in HS tissues and fibroblasts and confirmed that miR-143-3p inhibits HS formation by regulating the proliferation and apoptosis of human HSF [19]. Wei et al. found that miR-143-3p was downregulated in HS compared with normal skin tissue, and the overexpression of miR-143-3p inhibited the proliferation and invasion of HSF and promoted its apoptosis. They also confirmed that miR-143-3p played the above role by directly targeting Smad3 [20]. Besides, miR-92a-3p [21] was also involved in the development of various fibrotic diseases, but the correlation with keloid has not been reported.

The article "Identifying miRNAs Associated with the Progression of Keloid through mRNA-miRNA Network Analysis and Validating the Targets of miR-29a-3p in Keloid Fibroblasts" was published in 2022. Journal: Biomed Res Int.

Other target genes in the miRNA-mRNA network were also potentially involved in the development of keloid. For example, COL6A2 and COL6A3 jointly encode type VI collagen, and their mutation will lead to an autosomal dominant disease, namely Bethlem myopathy. James, Aralikatte, Edmar, Constanza et al. reported the formation of spontaneous keloid in patients with Bethlem myopathy, suggesting that there is a potential correlation between the imbalance of type VI collagen and the occurrence of keloid [22–25]. In addition, Georgios et al. found that type VI collagen was expressed in the extended edge of human keloid samples and confirmed that type VI collagen is a key regulator of dermal matrix assembly, composition, and fibroblast behavior and may play an important role in wound healing and tissue regeneration [26]. Periostin (POSTN) is a matricellular protein normally expressed in adult skin. Previous studies reported that POSTN was overexpressed in keloid and hypertrophic scars and increased POSTIN expression affects the proliferation, collagen synthesis, migration, and invasion of keloid fibroblasts under hypoxic conditions [27, 28].

In a word, the miRNA-mRNA network we constructed intuitively presents the regulatory effect of Hub miRNAs on Hub genes, effectively reveal the key genes and regulatory targets in the development of keloid, and lay the foundation for the development of new treatment schemes.

The current research mainly identifies the DEGs in keloid through high-throughput sequencing technology and bioinformatics analysis technology, to screen new therapeutic targets and potential biomarkers [7–9]. However, due to the different samples, different control groups, and small sample sizes, the sequencing results obtained from different studies are quite different and lack reliability. In this study, 6 datasets consisting of 20 keloid patients were screened from the GEO and ArrayExpress databases according to the inclusion and exclusion criteria. The samples and control groups were strictly controlled, and the sample size was expanded to a certain extent. GSE113619 and GSE113620 datasets were used as validation datasets to verify the expression levels of mRNA and miRNA, respectively, and RT-qPCR was used to verify the miRNA-mRNA network, which enhanced the reliability of the analysis results and reduced the false positive rate.

However, our research still has the following limitations: (1) there was no classified analysis of keloid patients with different races, different causes, and different parts; (2) focus on obtaining the most important genes and lack of attention to other genes; (3) the regulation of target genes by miRNA was predicted by ENCORI and has not been further verified by experiments; and (4) the potential target of miR-29a-3p has only been preliminarily verified, and more in-depth research is needed in in vivo and in vitro models.

The article "Identifying miRNAs Associated with the Progression of Keloid through mRNA-miRNA Network Analysis and Validating the Targets of miR-29a-3p in Keloid Fibroblasts" was published in 2022. Journal: Biomed Res Int.

## 5. Conclusions

In conclusion, DEGs between keloid and normal skin tissue were identified and functionally annotated through the analysis of gene expression data from multiple datasets. The miRNA-mRNA network was constructed, and the real central gene miR-29a-3p was screened. The potential target of miR-29a-3p was preliminarily verified, which provides a potential treatment option for the treatment of keloid.

## Figures and Tables

**Figure 1:** Flowchart of dataset selection.

**Figure 2:** The volcano plots of DEGs in GSE92566 (a), GSE83286 (b), GSE158395 (c), and GSE190626 (d) datasets.

**Figure 3:** 493 co-DEGs consisting of 318 co-up DEGs (a) and 175 co-down DEGs (b) exist in at least 3 discovery datasets.

**Figure 4:** GO analysis of 318 co-up DEGs (a) and 175 co-down DEGs (b).

**Figure 5:** KEGG analysis of 318 co-up DEGs (a) and 175 co-down DEGs (b).

**Figure 6:** PPI network of 493 co-DEGs.

**Figure 7:** Validation of the expression of Hub genes by GSE113619 dataset.

**Figure 8:** Validation of the expression of Hub miRNAs by GSE113620 dataset.

**Figure 9:** miRNA-mRNA network consisting of 15 miRNAs (3 downregulated and 12 upregulated) and 12 mRNAs (upregulated).

**Figure 10:** The relative expression of the miRNA-mRNA network was validated by RT-qPCR.

**Figure 11:** The relative expression of Hub genes when miR-29a-3p mimic or inhibitor was transfected into KFs.

**Figure 12:** Diagnostic value of COL1A1, COL1A2, COL3A1, COL5A1, and COL5A2 in keloid.

**Table 1:** Clinical specimen information.

Gender	Age (years)	Position	Etiology	Disease duration (years)
Female	55	Right forearm	—	7
Female	25	Right back	Folliculitis	3
Female	35	Right back	Folliculitis	8
Female	33	Chest	Acne	7
Female	41	Right auricle	Trauma	10
Male	39	Chest	—	5
Male	45	Chest	—	6
Male	12	Neck	Burns	10

**Table 2:** Primer sequences used for RT-qPCR.

Gene symbol	Primer sequences	
COL1A1	Forward	5′-CCCCTGGAAAGAATGGAGATG-3′
	Reverse	5′-TCCAAACCACTGAAACCTCTG-3′
COL1A2	Forward	5′-AGGACAAGAAACACGTCTGG-3′
	Reverse	5′-GGTGATGTTCTGAGAGGCATAG-3′
COL3A1	Forward	5′-GTGCACCTACTTCAAGCTCTAC-3′
	Reverse	5′-GCTTGAGGTTCTCGGGATTT-3′
COL5A1	Forward	5′-TCGCTTACAGAGTCACCAAAG-3′
	Reverse	5′-GTTGTAGATGGAGACCAGGAAG-3′
COL5A2	Forward	5′-AGCAAACCCATCCAGTGTAC-3′
	Reverse	5′-TGGCTGTATTAGGTGATTGGTG-3′
COL6A2	Forward	5′-TGAAACACGAAGCCTACGG-3′
	Reverse	5′-TCTCCCTGTCTTCCCTTCTG-3′
COL6A3	Forward	5′-CATTGGCTCTCACTGAAACAG-3′
	Reverse	5′-CCACAACCTCCATACCAGAATC-3′
COL11A1	Forward	5′-TTGGTGTTGAGGTTGGGAG-3′
	Reverse	5′-TTCTCCACGCTGATTGCTAC-3′
FBN1	Forward	5′-ACCCTATGCCAAGTTGATCC-3′
	Reverse	5′-ACTGACACTTGAATGACCCC-3′
GAPDH	Forward	5′-TCAACGACCACTTTGTCAAGCTCA-3′
	Reverse	5′-GCTGGTGGTCCAGGGGTCTTACT-3′

The article "Identifying miRNAs Associated with the Progression of Keloid through mRNA-miRNA Network Analysis and Validating the Targets of miR-29a-3p in Keloid Fibroblasts" was published in 2022. Journal: Biomed Res Int.

**Table 3:** The characteristics of the datasets included in the analysis.

GEO datasets	Library strategy	Cases	Overall design	Function in the analysis
GSE92566	Microarray	3 keloid patients	The transcriptional profile of biopsies from large chronic keloids, adjacent nonlesional skin (*n* = 3)	Discovery datasets for summarizing the significantly DEGs
GSE83286	Microarray	3 keloid patients	Microarray analysis was used to determine the expression profiles of lncRNAs and mRNAs between 3 pairs of earlobe keloid and normal specimens	
GSE158395	RNA-seq	3 keloid patients	The transcriptional profiling of lesional and nonlesional keloid skin	
GSE190626	RNA-seq	3 keloid patients	The transcriptional profiling of keloid tissue and adjacent normal tissues	
GSE113619	RNA-seq	8 keloid-prone individuals and 6 healthy individuals	3 mm punch biopsies of nonlesional upper outer buttock skin, followed by an additional 4 mm punch biopsy of the same site 6 weeks later (RNA-seq)	Validation dataset to validate the mRNA expression levels
GSE113620	Microarray	8 keloid-prone individuals and 6 healthy individuals	3 mm punch biopsies of nonlesional upper outer buttock skin, followed by an additional 4 mm punch biopsy of the same site 6 weeks later (miRNA)	Validation dataset to validate the miRNA expression levels
GSE188952	RNA-seq	4 keloid patients, 5 hypertrophic scars patients, and 3 normal scars patients	RNA-seq of normal scar, hypertrophic scar, and keloid	Evaluation of the diagnostic value of key genes in keloid

**Table 4:** 493 co-DEGs (318 co-up DEGs and 175 co-down DEGs).

Co-up DEGs (318)	PTN ST6GAL2 GREM1 F2RL2 ELN ARL4C TMEM200A FBLN7 TMEM176A KIF5C OAF CNPY4 TPBG TMEM176B PLAU LSAMP EDNRA GPR68 DNAH12 TDO2 ECM2 COL10A1 LAMP5 ADAMTS16 COL11A1 MFAP2 MDK ITGA10 GLIS3 THBS4 PAX1 ZNF469 PYCR1 GALNT5 TMEM92 RUNX2 PXDN AMPH MEG9 SULF2 NREP THY1 CADPS PCDH17 BGN DNM3OS CH25H TRO CASC15 GPX7 EPHB2 LINC01116 GLT8D2 CHPF COL8A1 CALU TRANK1 CSMD2 PDE1A DOK5 TTYH3 COL5A2 MS4A7 C2 FZD2 NID1 SUGCT BAG2 PRAF2 SLC41A2 ARHGEF25 PRDM6 MEG3 CLEC11A TPBGL CTHRC1 RFTN2 CALD1 THSD7A BICC1 EFEMP2 CHRD ARMC9 CRISPLD2 ADAMTS1 KHDRBS3 LAYN FIBIN ANTXR1 RRBP1 FBXL7 PPIC SH3RF3 SLC2A10 CREB3L1 NBL1 MX2 GPR4 TP53I3 NR2F1-AS1 ORAI2 C2orf27A SEMA6B MMP19 DZIP1 GRB10 THBS3 ATP8B3 DLG4 ATP10A LRRC15 MLLT11 GJA5 OAS2 SLC39A7 ZNF521 ZNF275 C11orf24 PDE7B BCL6B DPY19L3 SNHG18 MAGED1 NEK6 LPCAT1 SMARCA1 COL3A1 ENAH FAM229B NLGN2 PRSS23 ARPC1B LAMA2 SLFN11 COPZ2 CNTN4 DCLK2 SDK1 CTSK HTRA1 IGF2 TNFAIP6 THBS2 RYR2 PDGFRL TIMP1 TGFB1 ARHGAP28 ADAMTSL1 ARSB MSR1 DPP4 ITGBL1 ITGA4 TRAM2 MYO1B PODN TSHZ3 ST3GAL2 GFPT2 PDGFRB ADAMTS4 HIC1 TNC SCN1B SCARF2 RCN1 ADAM23 SLC36A1 HTRA3 PDIA5 CD276 IFI16 ADAMTS7 CYTL1 VOPP1 GLT8D1 CHST1 CARD6 PEAK1 SAMD9L P4HA3 SFRP4 CPXM1 SYNDIG1 COMP ADAM12 CILP2 COL14A1 OLFML2B ACAN ASPN SULF1 ADAMTS14 CDH11 GRIN2D PIEZO2 C1QTNF6 TNFSF4 PLAUR ADAMTS12 CHSY3 CGREF1 KDELR3 COL12A1 TMEM119 ALPK2 FKBP10 MMP14 FNDC1 LRRC17 SERPINH1 FAP VCAN HEY2 SGCD SORCS2 TGFB3 COL6A1 CERCAM MMP16 GXYLT2 RCN3 SPON1 NOX4 UCHL1 PCOLCE C1S ZFHX4 ROR2 COL5A1 NID2 ADAMTS6 POSTN KCNMA1 SFRP2 NNMT HMCN1 OGN IGDCC4 CHN1 ANGPTL2 GEM RHOBTB1 FMNL3 SSC5D COL1A1 NPTX2 SEC24D ISG15 FKBP14 GPX8 SEMA3A DACT1 ADAM19 RAB31 IKBIP SH3PXD2B FN1 ADAMTS2 COL6A2 PAPSS2 EDIL3 CHST11 PRR16 NRP2 LUM RNF144A BMP1 BEND6 SATB2 PLXDC1 GUCY1A2 FKBP7 MN1 MXRA8 SHOX2 NR2F1 FBN1 BNC2 LAMB1 CMTM3 HAPLN3 NRP1 PRRX1 AEBP1 OMD MARCKS NAV1 MAP4K4 COL16A1 OLFML3 SEC23A KCNE4 FKBP11 LOX MRC2 ALDH1L2 LRRC32 COL1A2 DCHS1 BCAT1 EPHA3 BASP1 RHOJ COL6A3 IL1R1 EVI2A ATP8B2 L3MBTL3 LOXL2 PGM3 SYTL2 STEAP1 TPST1 PRR5L FUCA2 MXRA5

Co-down DEGs (175)	VSIG10L SH3BGRL2 MATN4 HSD11B2 SCNN1G SLC14A1 KRT75 RHCG CHDH PLAG1 SPDEF MYBPC1 TMEM61 ESRRG EML2 KLK1 SUSD2 TRNP1 OCLN TPD52L1 SPIRE2 TBX3 FBXO32 ACSS2 SLC25A4 ADAMTSL3 SLC46A2 SYNGR1 CYP39A1 GLDN RRAGD USP54 ECHDC3 CHCHD10 COBL SORT1 LNX1 GCNT2 KRT77 C1orf226 SLC29A2 CDH22 PNPLA3 NRG2 ME1 CLYBL TMOD1 KRTCAP3 NEDD4L TMEM125 TST PLEKHG6 RASD1 GPRC5C CEACAM1 NNAT EPB41L4B SLC4A11 LIPH REEP6 CYP4X1 DNAH17 RNF128 ZG16B RAB3B CLDN8 RASSF10 SLC13A2 PLIN5 BEX2 CCL28 DLX4 DHCR7 KIAA0895 FOXC1 CHI3L1 JPH2 PAMR1 GPD1 SGCG HSD11B1 STK32A KCNQ4 SOX9 SAPCD2 HMGCS2 FAM189A2 MSMB RASD2 GPR12 CDA STAC2 ABTB2 SYNM MUCL1 CYP4F8 TNNI2 KCNMB1 SLC12A2 MGST1 BAMBI MAL ATP13A5 PADI2 ATP6V1B1 PPARGC1A KCNN4 CEACAM5 CLDN7 MYEOV PPP1R1A SHANK2 ELF3 KRT7 EPCAM ANXA3 KLRG2 G0S2 EDAR RHPN2 CNN1 CIDEC MMP7 GAL KRT18 YBX2 FA2H PRR15L PPP1R1B GABRP KRT19 ACTG2 THRSP TSPAN8 CEACAM6 PLIN4 SPRR4 CA6 KRT79 PLIN1 CLDN10 DNER SCGB2A2 ADIPOQ DCD SCGB1D2 PIP PRRG2 SRCIN1 HOXC13 TOB1 CADM4 FANCE CPEB3 PDCD4 GCHFR TFAP2B ATP1A1 PFKFB3 SLC25A23 EEF1A2 PANK1 RAP1GAP CHRM1 ELF5 SLC2A4 NCALD SH3D21 TMPRSS2 FMO5 ATP1B1 S100A1 KCNK5 AQP5 ATP6V0A4

The article "Identifying miRNAs Associated with the Progression of Keloid through mRNA-miRNA Network Analysis and Validating the Targets of miR-29a-3p in Keloid Fibroblasts" was published in 2022. Journal: Biomed Res Int.

**Table 5:** The top 20 genes ranked by different methods of Cytohubba.

	MCC	DMNC	MNC	Degree	EPC	Bottleneck	Eccentricity	Closeness	Radiality	Betweenness	Stress	Clustering coefficient
1	COL1A1	NID2	FN1	FN1	PDGFRB	FN1	FN1	FN1	FN1	FN1	FN1	FBLN7
2	COL1A2	COL8A1	COL1A1	COL1A1	FAP	DLG4	ANGPTL2	COL1A1	COL1A1	DLG4	COL1A1	LRRC32
3	COL3A1	THSD7A	COL1A2	COL1A2	GREM1	TGFB3	KRT18	COL1A2	COL1A2	COL1A1	DLG4	NNAT
4	COL5A1	COL14A1	COL3A1	COL3A1	LOXL2	PPARGC1A	NRP1	COL3A1	COL3A1	SOX9	SOX9	CEACAM1
5	COL6A1	NID1	POSTN	POSTN	LAMA2	RYR2	IGF2	BGN	BGN	BGN	COL1A2	IFI16
6	COL5A2	LOXL2	BGN	BGN	P4HA3	VCAN	PRRX1	POSTN	POSTN	PPARGC1A	BGN	OAS2
7	COL6A3	AEBP1	COL5A1	COL5A2	ITGA10	SCNN1G	EPHB2	COL5A2	COL5A2	KCNMA1	PPARGC1A	CYP39A1
8	LUM	ADAMTS16	COL5A2	COL5A1	ACAN	IGF2	DNER	COL5A1	SOX9	RUNX2	TGFB3	CHI3L1
9	BGN	LAMB1	FBN1	COL6A1	TIMP1	PDGFRB	PDGFRB	COL6A1	COL5A1	ADIPOQ	ADIPOQ	PLIN4
10	COL6A2	PCOLCE	COL6A1	FBN1	TGFB1	THY1	ANTXR1	FBN1	LOX	RYR2	ADAMTS4	CLDN8
11	COL12A1	P4HA3	THBS2	THBS2	COMP	POSTN	FKBP10	SOX9	TGFB3	COL1A2	COL5A1	MS4A7
12	COL11A1	SPON1	COL6A2	COL6A2	COL1A1	COL6A3	MDK	COL6A2	ELN	COL5A1	FKBP10	SCGB1D2
13	COL16A1	PRRX1	LUM	LUM	TGFB3	SOX9	OCLN	ELN	THY1	THY1	COL6A1	SEMA6B
14	POSTN	COL16A1	ACAN	ADAMTS2	SOX9	SERPINH1	FAP	LUM	TGFB1	ADAMTS4	COL3A1	MSR1
15	FBN1	MFAP2	COL6A3	COL6A3	ADAMTS2	EPHB2	FBLN7	LOX	FBN1	TGFB3	ADAMTS2	PFKFB3
16	PCOLCE	LAMA2	ELN	ACAN	MMP7	KCNMA1	SFRP4	COL6A3	COL6A1	FKBP10	RYR2	MYO1B
17	COL14A1	ADAMTSL3	ADAMTS2	ELN	OGN	NOX4	EPCAM	THBS2	TIMP1	COL6A1	RUNX2	THSD7A
18	FN1	COL12A1	COL11A1	COL11A1	NID1	RUNX2	PLAUR	ACAN	COL6A2	COL3A1	FA2H	PYCR1
19	THBS2	COL11A1	VCAN	VCAN	VCAN	OCLN	GREM1	TGFB3	LUM	FA2H	THY1	DACT1
20	SERPINH1	LUM	LOX	ADAMTS4	LUM	ADAMTS4	CHSY3	COL11A1	COL6A3	EPHB2	TGFB1	AEBP1

## Data Availability

Data are available from GSE92566 (https://www.ncbi.nlm.nih.gov/geo/query/acc.cgi?acc=GSE92566), GSE83286 (https://www.ncbi.nlm.nih.gov/geo/query/acc.cgi?acc=GSE83286), GSE158395 (https://www.ncbi.nlm.nih.gov/geo/query/acc.cgi?acc=GSE158395), GSE190626 (https://www.ncbi.nlm.nih.gov/geo/query/acc.cgi?acc=GSE190626), GSE113619 (https://www.ncbi.nlm.nih.gov/geo/query/acc.cgi?acc=GSE113619), GSE113620 (https://www.ncbi.nlm.nih.gov/geo/query/acc.cgi?acc=GSE113620), GSE188952 (https://www.ncbi.nlm.nih.gov/geo/query/acc.cgi?acc=GSE188952).
